The article "β-glucan administration improves growth performance and gut health in New Zealand White and APRI rabbits with different breed responses" was retracted in 2024. Reasons: errors in the data; duplicated images; overlap with earlier publications; unreliable data.

# β-glucan administration improves growth performance and gut health in New Zealand White and APRI rabbits with different breed responses

**DOI:** 10.1371/journal.pone.0234076

**Published:** 2020-06-10

**Authors:** Mahmoud M. Abo Ghanima, Ayman H. Abd El-Aziz, Ahmed E. Noreldin, Mustafa S. Atta, Shaker A. Mousa, Ali H. El-Far

**Affiliations:** 1 Department of Animal Husbandry and Animal Wealth Development, Faculty of Veterinary Medicine, Damanhour University, Damanhour, Egypt; 2 Department of Histology and Cytology, Faculty of Veterinary Medicine, Damanhour University, Damanhour, Egypt; 3 Department of Physiology, Faculty of Veterinary Medicine, Kafrelsheikh University, Kafrelsheikh, Egypt; 4 Pharmaceutical Research Institute, Albany College of Pharmacy and Health Sciences, Rensselaer, NY, United States of America; 5 Department of Biochemistry, Faculty of Veterinary Medicine, Damanhour University, Damanhour, Egypt; INIA, SPAIN

## Abstract

This study investigated the effects of oral administration of β-glucan 1,3 (pharmaceutical grade 10%) on growth performance and carcass traits in two breeds of weanling rabbits adapted to survive in Egypt, New Zealand White (NZW) and Animal Production Research Institute (APRI) rabbits, with special attention to relative mRNA expression of interleukins and antioxidant enzyme genes, biochemical, and histological alterations. Oral administration of β-glucan with doses 0.25 and 0.5 ml per one-liter of drinking water significantly accelerated body weight gain (BWG) in both rabbits’ breeds, reduced total feed consumption (FC), and reduced feed conversion ratio (FCR), especially the 0.5 ml per one-liter dose in both rabbit breeds. There are remarkable differences in all the growth performance traits due to breed effect. The interaction effect between β-glucan and breed significantly improved BWG, FC, and FCR. There were non-significant differences in all carcass traits studied due to oral administration of β-glucan with both doses, except in dressing percentages. The highest of the dressing percentages were observed at doses 0.25 ml per one-liter (51%) and 0.5 ml per one-liter (52%) compared with control (50%). Our findings show significant variations in the final BW, total daily gain, feed consumption, and total feed conversion ratio between NZW and APRI rabbits. Absence of significant differences in the hot carcass weight and dressing percentage between the genetic groups had been reported in this study. Supplementing NZW and APRI rabbits with β-glucan increased blood total protein and globulin. The duodenal villi dimensions, splenic lymphoid diameter, muscular fiber diameter, and muscular glycogen areas were significantly increased by β-glucan administration. Expression of intestinal interleukin-18 (*IL-18*) in NZW rabbits treated with 0.25 and 0.5 doses of β-glucan was significantly upregulated and enhanced the immune response. β-glucan upregulated the expression of intestinal *occludin* mRNA particularly at dose 0.5 β-glucan as well as upregulated intestinal superoxide dismutase 1 (*SOD1*) and glutathione peroxidase 1 (*GPx1*), which modulates anti-inflammatory and antioxidant properties. In conclusion, oral administration of β-glucan at a dose of 0.25 or 0.5 ml per one-liter drinking water provided beneficial effects in the growth performance and health status of rabbits.

## Introduction

Rabbits meat production is a practical solutions to the growing protein shortage in developing countries [1]. In many European and North African countries, including Egypt, meat is consumed routinely and its production plays a major role in most of those countries' economies [2]. To help resolve the global protein shortage problem, production of rabbits is an appropriate task due to high fertility, low investment costs, a short interval between generations, and the ability to use various forages [3]. Rabbit meats are also highly digestible, delicious, and low-calorie foods that nutritionists often recommend over other meats [4] because rabbit meat is about 20% proteins, unsaturated fatty acids, potassium, phosphorus, and magnesium along with low contents of fat, cholesterol, and sodium [5].

The European Union prohibition of the use of antibiotic growth promoters led to research for various natural feed additives rather than food antibiotics including probiotics, prebiotics, enzymes, and organic acids [6]. A natural feed additive is β-1,3–1,6-glucan, the structural constituent that is present in the cell wall of yeast, fungi, and certain bacteria [7]. β-1,3–1,6-glucan can be supplied as alternate feed additive orally and is absorbed by intestinal cells and intestinal lymphoid tissue cells into the gastrointestinal tract, stimulating molecular and humoral immune reaction cells [8]. Advances were noted in immunity by supplementing β-1,3–1,6-glucan in rabbits [9] chicken [10], swine [11], and horse [12].

The current research was therefore carried out to explore the impacts of oral administration on the growth and carcass characteristics, with specific attention paid to their molecular, biochemical, and histopathological changes, in New Zealand White (NZW) and Animal Production Research Institute (APRI) rabbits, two races of weaning rabbits adapted to survive in Egypt.

## Materials and methods

### Ethical statement

The research was endorsed by the Faculty of Veterinary Medicine (Damanhour University, Egypt), committee of Local Experimental Animal Care. During the experiment, all precautions were taken to reduce the animal suffering.

### Animals, management, and the experimental design

A new maternal line (APRI) established from Egyptian Baladi Red (BR) and a Spanish line (V) rabbits was started in 2002 at the Sakha experimental rabbitry, Animal Production Research Institute, Agricultural Research Center, Ministry of Agriculture, Egypt. The APRI line was established by crossing Baladi Red bucks with V line does to produce F1 (½B½V) stock, followed by two generations of inter se matings to achieve performance stability. Rabbits of both breeds at the 6^th^ week of age and 680±40 g body weight were allotted randomly into 6 groups (20 rabbits per each). This experiment was carried out at a private farm on these 120 weaned male rabbits of 6 weeks of age (680±40 g live body weight). Animals were allotted into a completely randomized design in a 2 × 3 factorial arrangement (two breeds: NZW and APRI, and three levels of β-glucan (βG): 0 (control), 0.25, and 0.5 ml per one-liter drinking water).

Rabbits were reared in a semi-closed rabbitry of 180 m^2^ (6 m width and 30 m length) with wire-netted windows in eastern and western sides for natural ventilation. Windows were oriented with an elevation of 160 cm from the floor, which was concrete with moderate slope to middle to facilitate drainage of water and waste liquids towards large gutters to the outside. During cold, windy weather and at night the windows were closed for protection from severe atmosphere.

Rabbits were housed in galvanized wire batteries with standard dimensions (60 x 35 x 35 cm). All cages were supplied with galvanized-steel feeding hoppers and automatic drinkers (nipples). Rabbits were identified by plastic ear tags. Fresh water was offered *ad libitum*. Rabbits were fed on a standard pelleted ration offered *ad libitum* twice daily at 8 am and 2 pm. The pellets were 1 cm length and 0.4 cm diameter. Rabbit cages were regularly cleaned and disinfected. Urine and feces dropped beneath the batteries were removed every day in the morning.

Rabbits from each breed were allocated into 3 groups (20 rabbits each) with one group considered as a control. The treated groups received β-glucan 1,3 pharmaceutical grade 10% concentration at a dose of either 0.25 ml or 0.5 ml per one-liter of drinking water for 3 successive days each week. Each individual rabbit in 0.25 ml β-glucan-treated group was supplemented with 233.25 mg of β-glucan during 10-week experimental period, while in 0.5 ml β-glucan-treated group each rabbit was supplemented with 466.5 mg of β-glucan. Modulin Plus^®^ (Micro-Biotech Company, Miami, FL, USA) was used as a source of β-glucan 1,3 pharmaceutical grade (10%).

### Experimental diet

The basal experimental diet was formulated following the NRC [13] and de Blas and Mateos [14] recommendations and then pelleted to satisfy the nutrient requirements of rabbits (Table 1). Ingredients needed for formulation of the experimental diets were finely ground by using hammer mill screen size 3.0 mm, then weighing of different ingredients at required amount for the experimental diets, thoroughly mixed and pelleted (3.5 mm size).

**Table 1:** Ingredients and chemical composition (%) of the basal diet.

Ingredients	Percentages
Yellow corn	9.5
Soybean meal 44%	15.0
Wheat bran	17.0
Barley	21.7
B. Hay	34.5
Dicalcium phosphate*	1.2
Ground limestone**	0.25
DL-Methionine	0.05
Common salt	0.5
Vitamin + Mineral premix***	0.3
Total	100
**Chemical composition of the basal diet**	
Dry matter	87.8
Moisture	12.2
Crude protein	17.9
Crude fiber	13.75
Ether extract	3.6
Nitrogen-free extract^ɸ^	42.75
Ash	9.8
DE (kcal/kg) ^ɸɸ^	2677.97

* Dicalcium phosphate contains 20% phosphorus and 25% calcium

** Limestone: contains 34% calcium

*** Every 1 kg of ration contains the following vitamins and minerals: vitamin A– 12000 IU; vitamin D3–900 IU; vitamin E– 50 mg; vitamin k3–2 mg; vitamin B1–2 mg; vitamin B2–6 mg; vitamin B6–2 mg; vitamin B12–0.01 mg; biotin– 0.2 mg; pantothenic– 20 mg; niacin– 50 mg; folic acid– 5 mg; manganese– 8.5 mg; zinc– 70 mg; iron– 75 mg; copper– 5 mg; iodine– 0.75 mg; selenium– 0.1 mg.

^ɸ^ NFE was calculated by difference = 100 –(moisture % + CP% + EE% + CF% + Ash %).

^ɸɸ^ Digestible energy (DE) was calculated according to values given in the feed composition tables of the NRC [13].

### Growth performance traits

Rabbits were individually weighed at the beginning (6^th^ week) and at the 16^th^ week of age, then daily weight gain was calculated during the whole period. Weighing was done in the early morning before rabbits received any feed or water. Feed consumption per rabbit was recorded daily. Residues and wasted feed were weighed daily and then subtracted from the offered amounts to obtain the actual accumulated feed consumed, and then the feed conversion ratio (FCR) was calculated. Also, body weight (BW), body weight gain (BWG), and total feed conversion (FC) were determined [15].

### Carcass traits

At the 16^th^ week, 3 representative rabbits from each group were randomly taken to estimate the carcass traits. Rabbits were fasted for approximately 6 hours before sacrifice and then individually weighed. Carcass was eviscerated after skinning, and giblets (liver, heart, and kidneys) were removed and weighed to determine the dressed weight and the dressing percentage. All data were recorded as percentage to the live body weight [16].

Dressing percentage was calculated as (hot carcass weight × 100/fasted weight). Carcass was separated for the following three cuts: (1) two fore legs (including thoracic insertion muscles), (2) loin (including the abdominal wall and the ribs after the 7^th^ thoracic rib), and (3) hind legs (including the sacral bone and the lumber vertebra after the 6^th^ lumber vertebra).

### Biochemical assessments

After sacrifice, blood samples (*n* = 5 for each group) were collected and then tubes were left in slope position until serum samples were separated through centrifugation at 1000 ×*g* for 20 minutes. The collected sera were subjected to biochemical analyses.

Serum total protein, albumin, alanine aminotransferase (ALT), aspartate aminotransferase (AST), creatinine, and urea were determined using commercial kits according to the manufacturers’ instructions (Bio-diagnostic, Giza, Egypt). Serum globulin concentration was calculated by the difference between total protein and albumin, and the albumin/globulin ratios were calculated.

### Histomorphometry

Five samples from five different rabbits of each group of one cm in length were sliced from dueodenum, spleen, and pectoral muscle preserved in 4% paraformaldehyde dissolved in PBS. Then, tissues were prepared using the standard histological technique including dehydration with ascending percentage of ethanol until reaching 100% ethanol. Then, cleared in xylene and melted paraffin ended by embedding in paraffin wax at 65°C. The paraffin blocks were sectioned at 4μm thickness using a microtome, then these sections were stained with Hematoxylin and Eosin (H&E) and for periodic acid schiff (PAS) according to the method of Bancroft and Layton [17].

From each intestinal segment, three sections were used (one section from serial 10 sections). From every section, 5 complete villi having perfect orientation and intact lamina propria were selected indiscriminately for inspection. Therefore, an average of 15 values were obtained for each intestinal sample. Slides were examined under a light microscope (Leica DM500, Leica, Germany) at 4X magnification, supported with a digital camera (Leica EC3). Images were analyzed with an image processing system photo analyzer (Image J; v1.46r, NIH, Bethesda, MD, USA) as described by Schneider et al (2012). The variables calculated for histomorphological modulations were crypt depth (CD), villus height (VH), villus width (VW), and villus height to crypts depth ratio (VH: CD) according to the method of Saeed et al [18] and Kiczorowska et al [19].

Well-oriented germinal center areas in the spleen were combined together and were noted as a percentage of the total field of view at 4X magnification using a Leica light microscope (Madej et al., 2015) and measured as optical denisty of splenic white pulp by (Image J). Later the average of 3 sections values was determined.

Cross dissections of pectoral muscle were processed, sectioned, and stained for quantification of mean fiber cross-sectional area as previously described Heywood et al [20], and the glycogen area was evaluated according to the protocol of Prats et al [21]. Light photomicrographs at 40X magnification were taken using a Leica light microscope and images were analyzed using Image J.

### Assessment of gene expression

Total RNA was obtained from the samples (*n* = 5 for each group) using easy-RED Total RNA Extraction Kits (iNtRON Biotechnology, Inc., Korea) as directed by the manufacturer. Agarose gel electrophoresis was used to check the integrity of RNA, and a NanoDrop spectrophotometer was used to analyze the quantities and purities of the samples. First-strand cDNA was obtained using a kit for HiSenScript cDNA (iNtRON Biotechnology, Inc., Korea). Specific primers were used to amplify chosen genes with GAPDH as a housekeeping gene that was stable among the sample groups (Table 2). The mRNA expression was performed using a Stratagene MX3005P real-time PCR (Agilent Technologies, CA, USA) and TOPreal^TM^ PreMIX SYBR Green qPCR master blend (Enzynomics, Daejeon, Republic of Korea) following the suggestions of the manufacturer. MxPro QPCR Software was used. The relative concentrations of gene expression were assessed using the 2^−ΔΔct^ technique as outlined in Pfaffl [22].

**Table 2:** Primers for gene expression by RT-PCR.

Genes	Primer sequence (5’→3’)	Accession No.
Interleukin-4 (*IL-4*)	F: CCCAAGAACACAACCGAGAG	NM_001163177.1
	R: AGTCTGTCTGGCTTCCTTCC	
Interleukin-6 (*IL-6*)	F: TCCAGGAGCCCGACTATGAA	NM_001082064.2
	R: TCGTCACTCCTGAACTTGGC	
Interleukin-10 (*IL-10*)	F: AGAACCACAGTCCAGCCATC	NM_001082045.1
	R: GCTTTGTAGACGCCTTCCTC	
Interleukin-18 (*IL-18*)	F: AGAAAATGCACCCCAGACCA	NM_001122940.1
	R: TCTTTCTGTCCTGCGAGATGT	
Interleukin-1β (*IL-1β*)	F: CCCCAACCGTTACCCAAAGA	NM_001082201.1
	R: GGGAACTGGGCAGACTCAAA	
Inducible nitric oxide synthase (*iNOS*)	F: CTCCGAGTACAAAGGGCTCC	XM_017349096.1
	R: CCTTGCGGACCATCTCCTG	
Interferon-γ (*IFN-γ*)	F: TCTTGGGTTCTTACGGCTGT	NM_001081991.1
	R: TGTTGTCACTCTCCTCTTTCCA	
Superoxide dismutase 1 (*SOD1*)	F: GCAGGCCCTCACTTTAATCC	NM_001082627.2
	R: CCTTTGCCCAAGTCGTCTTC	
Glutathione peroxidase 1 (*GPx1*)	F: GCCCAGTCTGTGTACTCCTT	NM_001085444.1
	R: CGTTCTCCTGATGCCCAAAC	
*Occludin*	F: TGCTTTTGTCTTACTGTTTACATGC	GBCI01075279.1
	R: GGCACAGCACCCAGAATAGT	
Glyceraldehyde 3-phosphate dehydrogenase (*GAPDH*)	F: TGTTTGTGATGGGCGTGAA	NM_001082253.1
	R: CCTCCACAATGCCGAAGT	

### Statistical analysis

The body weight data were normally distributed and subjected to statistical analysis using Two-way analysis of co-variance for initial body weight data; the general linear model (GLM) of the SAS program (SAS Institute, SAS^®^ 2009). The following model was fitted: Yijkl = μ + Wi + Sj+ Ek+ SEjk+ eijKl, where Yijkl = observed value of the concerned treatment, μ = observed mean for the concerned treatment, Wi = effect due to covariance of the initial weight, Sj = effect due to breed, Ek = effect due to β-glucan, SEjk = interaction effect due to breed and β-glucan, and eijkl = the error related to individual observation. While, the weight gain, feed consumption and feed conversion data were normally distributed and subjected to statistical analysis using Two-way analysis of variance for initial body weight data; the general linear model (GLM) of the SAS program (SAS Institute, SAS^®^ 2009). The following model was fitted: Yijk = μ +Si+ Ej+ SEij+ eijK, where Yijk = observed value of the concerned treatment, μ = observed mean for the concerned treatment, Si = effect due to breed, Ej = effect due to β-glucan, SEij = interaction effect due to breed and β-glucan, and eijk = the error related to individual observation. Differences between means were tested with Duncan's multiple range test at the level of α = 0.05 [23]. The percentages of the studied traits were transformed to Arcsine values and then re-transformed to the original values after analysis. Statistical analysis of gene expression data was done with one-way ANOVA and Tukey's post hoc test for multiple comparisons using with GraphPad prism 5 (San Diego, CA, USA).

## Results

### Growth performance

Results of growth performance (BW, BWG, FC, and FCR) are presented in Table 3. Oral administration of β-glucan at doses 0.25 and 0.5 ml per one-liter drinking water significantly (*P* < 0.05) accelerated BWG in rabbits and reduced FCR in comparison with control. The 0.5 ml per one-liter drinking water β-glucan administration was the best dose for rabbits. There is a remarkable difference in all growth performance traits due to breed effect. The interaction effect between β-glucan and breed was significant on BWG, FC, and FCR and the highest gain and the lowest FCR were noticed in each breed when interacted with β-glucan (Table 3).

**Table 3:** Growth performance of rabbits as affected by breed and β-glucan administration.

Items		Final body weight (g)	Body weight gain (g)	Total feed consumption (g)	Feed conversion ratio (g feed/g gain)
**Breed effect**					
**NZW**		2598.84 ^a^	1819.00 ^a^	5396.33 ^b^	3.155 ^b^
**APRI**		2383.16 ^b^	1726.00 ^b^	6072.33 ^a^	3.375 ^a^
**SEM**		4.86	8.47	0.289	0.016
**P value**		0.001	0.001	0.001	0.001
**β-glucan administration**					
**βG_0.25_**		2479.71 ^b^	1769.50 ^b^	5718.00 ^b^	3.230 ^b^
**βG_0.5_**		2672.97 ^a^	1939.00 ^a^	5422.50 ^c^	2.794 ^c^
**Control**		2320.31 ^c^	1609.00 ^c^	6062.50 ^a^	3.770 ^a^
**SEM**		4.86	8.47	0.289	0.016
**P value**		0.001	0.001	0.001	0.001
**Breed × treatment interactions**					
**NZW**	Control	2255.05 ^f^	1599.00 ^d^	5853.00 ^c^	3.664 ^b^
	βG_0.25_	2345.84 ^e^	1692.00 ^c^	5263.00 ^e^	3.112 ^d^
	βG_0.5_	2548.58 ^c^	1887.00 ^b^	5073.00 ^f^	2.688 ^f^
**APRI**	Control	2385.57 ^d^	1619.00 ^d^	6272.00 ^a^	3.876 ^a^
	βG_0.25_	2613.57 ^b^	1847.00 ^b^	6173.00 ^b^	3.348 ^c^
	βG_0.5_	2797.36 ^a^	1991.00 ^a^	5772.00 ^d^	2.900 ^e^
**SEM**		4.86	8.47	0.289	0.001
***P* value**		0.001	0.001	0.001	0.001

Means within each column for each division with no common superscript letters are significantly different (*P* < 0.05).

SEM = standard error of means. βG = β-glucan

### Carcass traits

Findings of carcass traits showed non-significant differences in all carcass traits studied for oral administration of β-glucan, breed, and their interaction (Table 4), except in forequarters, hindquarters, and dressing percentages (*P* < 0.05) due to the interaction between β-glucan and breed. The highest percentages of forequarters, hindquarters, and dressing percentages were obtained from NZW when administered with 0.5% β-glucan (33.2%, 41.9%, and 52.2%, respectively).

**Table 4:** Carcass traits of rabbits as affected by breed and β-glucan administration (%).

Items		Forequarter	Loin	Hindquarter	Giblets	Dressing
Breed						
NZW		0.327	0.282	0.400	0.056	0.513
APRI		0.325	0.272	0.399	0.050	0.510
SEM		0.004	0.004	0.003	0.003	0.002
*P* value		0.81	0.19	0.76	0.25	0.38
β-glucan treatment						
βG_0.25_		0.325	0.280	0.402	0.056	0.51 ^a^
βG_0.5_		0.332	0.281	0.405	0.051	0.52 ^a^
Control		0.322	0.269	0.391	0.050	0.50 ^b^
SEM		0.004	0.004	0.003	0.003	0.002
*P* value		0.52	0.32	0.13	0.58	0.002
Breed × treatment interactions						
NZW	Control	0.320 ^a^	0.270	0.383 ^b^	0.055	0.504 ^b^
	βG_0.25_	0.329 ^a^	0.280	0.400 ^ab^	0.056	0.514 ^ab^
	βG_0.5_	0.332 ^a^	0.295	0.419 ^a^	0.057	0.522 ^a^
APRI	Control	0.315 ^b^	0.267	0.392 ^b^	0.045	0.500 ^b^
	βG_0.25_	0.317 ^ab^	0.281	0.399 ^ab^	0.048	0.510 ^ab^
	βG_0.5_	0.344 ^a^	0.268	0.405 ^ab^	0.056	0.520 ^a^
SEM		0.004	0.004	0.003	0.003	0.002
*P* value		0.05	0.21	0.02	0.71	0.05

Means within each column for each division with no common superscript letters are significantly different (*P* < 0.05).

### Biochemical analyses

Administrating rabbits with β-glucan at a dose 0.5 ml per one-liter drinking water increased blood total protein and globulin values (Table 5). β-glucan significantly increased uric acid in comparison with control, while urea and creatinine levels were non-significantly changed

**Table 5:** Biochemical parameters of rabbits as affected by breed and β-glucan administration.

Items		TP	Albumin	Globulin	ALT	AST	Uric acid	Urea	Creatinine	A/G Ratio
Breed										
NZW		6.03	3.42	2.60	25.15	13.36	2.69 ^b^	24.59	0.84	1.39
APRI		6.27	3.55	2.72	22.39	11.71	3.02 ^a^	27.80	0.86	1.52
SEM		0.22	0.13	0.17	1.03	0.69	0.05	1.4	0.02	0.11
*P* value		0.58	0.64	0.73	0.19	0.24	0.004	0.07	0.53	0.57
β-glucan treatment										
βG0.25 6.05 3.29 2.73 20.59 12.61 3.04 ^a^ 29.59 0.85 1.32										
βG_0.5_		6.34	3.44	2.90	25.91	11.38	3.04 ^a^	24.62	0.86	1.31
Control		6.08	3.72	2.35	24.82	13.61	2.49 ^b^	27.38	0.84	1.76
SEM		0.22	0.13	0.17	1.03	0.69	0.05	1.4	0.02	0.11
*P* value		0.82	0.43	0.42	0.11	0.44	0.001	0.36	0.92	0.20
Breed × treatment interactions										
NZW	Control	5.92	3.11	2.23	20.25 ^b^	15.14	2.28 ^c^	25.77	0.83	1.74
	βG_0.25_	5.93	3.69	2.80	21.09 ^b^	11.97	2.96 ^ab^	28.23	0.86	1.15
	βG_0.5_	6.24	3.47	2.78	34.11 ^a^	12.97	2.84 ^ab^	19.78	0.84	1.30
APRI	Control	6.24	3.42	2.48	29.39 ^a^	12.07	2.70 ^b^	28.99	0.88	1.78
	βG_0.25_	6.13	3.46	2.66	20.09 ^b^	13.26	3.12 ^a^	30.94	0.86	1.48
	βG_0.5_	6.45	3.76	3.02	17.71 ^b^	9.79	3.23 ^a^	29.45	0.84	1.31
SEM		0.22	0.13	0.17	1.03	0.69	0.05	1.4	0.02	0.11
*P*value		0.98	0.79	0.81	0.001	0.40	0.001	0.27	0.954	0.54

Means within each column for each division with no common superscript letters are significantly different (*P* < 0.05).

SEM = standard error of the mean.

### Histomorphometry

Mucosal histomorphometric studies revealed significantly (*P* <0.05) higher VH in duodenum of groups treated with 0.5% β-glucan compared with control (Table 6) and (Fig 1). Moreover, higher VH:CD ratio was observed in duodenum of these groups. Furthermore, the number of infiltrated lymphocytes into the intestinal epithelium increased significantly in groups administered with 0.25% and 0.5% β-glucan compared with control (Table 6, Fig 2) with highest values in 0.5% β-glucan.

**Fig 1:** Light micrographs of duodenum revealing the effect of different doses of β glucan; control, 0.25 g β glucan (βG_0.25_), 0.5 g β glucan (βG_0.5_) on the two rabbit species; New Zealand White (NZW) and APRI rabbits were represented in (A to C) and from (D to F), respectively. The micrographs showing the increasing in the villi height (VH) from (A to C) and from (D to F). Villi (arrowheads), Brunner’s gland (arrows). PAS stain. *Scale bar* is 400 μm.

**Fig 2:** Light micrographs of duodenum showing the effect of different doses of β glucan; control, 0.25 g β glucan (βG_0.25_), 0.5 g β glucan (βG_0.5_) on the two rabbit species; New Zealand White (NZW) and APRI rabbits were represented in (A to C) and from (D to F), respectively. The micrographs revealing the different epithelial lymphocytic infiltration from (A to C) and from (D to F). Lymphocytes (arrowheads) and goblet cells (arrows). PAS stain. *Scale bar* is 50 μm.

**Table 6:** Histomorphometric changes of rabbits’ duodenum as affected by breed and β-glucan administration (μm).

Items		Villus height	Villus width	Crypt depth	VH/CD	No. of lymphocytes/villi
Breed						
NZW		877.89 ^a^	118.51 ^a^	105.78	9.02	95.778
APRI		762.83 ^b^	93.39 ^b^	110.98	7.31	99.556
SEM		18.06	3.78	5.17	0.454	1.155
*P* value		0.004	0.002	0.647	0.072	0.128
β-glucan treatment						
βG_0.25_ 785.03 ^b^ 106.60 104.25 8.29 89.500 ^b^						
βG_0.5_		930.89 ^a^	106.44	111.38	8.94	126.00 ^a^
Control		745.15 ^b^	103.30	109.52	7.25	77.500 ^c^
SEM		18.06	3.78	5.17	0.454	1.155
*P* value		0.001	0.925	0.863	0.329	0.001
Breed × treatment interactions						
NZW	Control	801.19 ^bcd^	121.36 ^a^	112.16	7.57	73.333 ^c^
	βG_0.25_	847.94 ^bc^	127.29 ^a^	100.07	9.60	88.333 ^b^
	βG_0.5_	984.52 ^a^	106.86 ^ab^	105.11	9.86	125.667 ^a^
APRI	Control	689.11 ^d^	85.23 ^b^	106.87	6.93	81.667 ^bc^
	βG_0.25_	722.11 ^cd^	85.92 ^b^	108.42	6.98	90.667 ^b^
	βG_0.5_	877.27 ^ab^	106.01 ^ab^	117.65	8.02	126.333 ^a^
SEM		18.06	3.78	5.17	0.454	1.155
*P* value		0.001	0.015	0.949	0.296	0.001

Means within each column for each division with no common superscript letters are significantly different (*P* < 0.05).

VH/CD = Villus height/Crypt depth

Germinal center areas of spleen in groups administered with 0.25% and 0.5% β glucan increased (*P* < 0.05) compared with control (Table 7, Fig 3).

**Fig 3:** Light micrographs of spleen showing the effect of different doses of β glucan; control, 0.25 g β glucan (βG_0.25_), 0.5 g β glucan (βG_0.5_) on the two rabbit species; New Zealand White (NZW) and APRI rabbits were represented in (A to C) and from (D to F), respectively. The micrographs revealing the increasing in the whole white pulp areas and the lymphoid nodules (arrows) diameter from (A to C) and from (D to F). H and E stain. *Scale bar* is 400 μm.

**Table 7:** Averages of total splenic white pulp areas/ 3 mm^2^.

Items		Total splenic white pulp area
Breed		
NZW		44811.79 ^a^
APRI		30146.46 ^b^
SEM		1869.503
*P* value		0.002
β-glucan treatment		
βG_0.25_		45430.136 ^a^
βG_0.5_		40873.803 ^a^
Control		26133.440 ^b^
SEM		1869.503
*P* value		0.003
Breed × treatment interactions		
NZW	Control	34570.902 ^b^
	βG_0.25_	60290.571 ^a^
	βG_0.5_	39573.901 ^b^
APRI	Control	17695.979 ^c^
	βG_0.25_	30569.700 ^bc^
	βG_0.5_	42173.704 ^b^
SEM		1869.503
*P* value		0.001

Means within each column for each division with no common superscript letters are significantly different (*P* < 0.05).

The mean fiber cross-sectional area of pectoral muscles and the glycogen areas were significantly improved in groups administered with 0.25% and 0.5% β-glucan (Table 8, Fig 4).

**Fig 4:** Light micrographs of muscle showing the effect of different doses of β glucan; control, 0.25 g β glucan (βG_0.25_), 0.5 g β glucan (βG_0.5_) on the two rabbit species; New Zealand White (NZW) and APRI rabbits were represented in (A to C) and from (D to F), respectively. The micrographs revealing the different glycogen content and muscle fiber cross-sectional area from (A to C) and from (D to F). Low glycogen muscle fibers (arrowheads) and high glycogen muscle fibers (arrows). PAS stain. *Scale bar* is 50 μm.

**Table 8:** Mean of muscle fiber cross-sectional area (μm^2^) and glycogen area/300 μm^2^.

Items		Muscle fiber cross-sectional area	Glycogen area
Breed			
NZW		2330.79 ^a^	728.10 ^a^
APRI		2048.90 ^b^	454.11 ^b^
SEM		62.56	54.06
*P* value		0.02	0.02
β-glucan treatment			
βG_0.25_ 2257.75 ^b^			762.97 ^a^
βG_0.5_		2672.75 ^a^	837.75 ^a^
Control		1639.53 ^c^	172.88 ^b^
SEM		62.56	54.06
*P* value		0.01	0.01
Breed × treatment interactions			
NZW	Control	1775.40 ^bc^	108.45 ^c^
	βG_0.25_	2502.11 ^a^	1099.70 ^a^
	βG_0.5_	2714.86 ^a^	976.14 ^a^
APRI	Control	1503.65 ^c^	237.30 ^c^
	βG_0.25_	2013.40 ^b^	425.64 ^bc^
	βG_0.5_	2629.66 ^a^	699.37 ^ab^
SEM		62.56	54.06
*P* value		0.01	0.01

Means within each column for each division with no common superscript letters are significantly different (*P* < 0.05).

### Gene expression assessment

In comparison with the control group, the expressions of intestinal interleukin-18 (*IL-18*) (Fig 5C) in NZW rabbits administered with 0.25 and 0.5 β-glucan were substantially upregulated. However, in separate treatment groups, there is no important impact on the expression of intestinal *IL-4*, *IL-10*, and interferon-γ (*IFN-γ*) (Fig 1A, 1B and 1D). Rabbits in NZW+βG_0.25_ and NZW+βG_0.5_ groups displayed significant upregulations (*P* < 0.01) in the expression of intestinal superoxide dismutase 1 (*SOD1*) (Fig 1E) in relation to the control group. In addition, 0.5 β-glucan treated group demonstrated significant upregulation (*P* < 0.001) of expression of intestinal glutathione peroxidase 1 (GPx1) (Fig 5F) compared with the other group. In addition, the NZW+βG_0.5_ group showed significant increases (*P* < 0.05) in intestinal *occludin* expression compared with the other groups (Fig 5G). NZW rabbit's mRNA expression of splenic *IL-1β*, *IL-6*, and inducible nitric oxide synthase (*iNOS*) shows no important distinction compared with control (Fig 6A, 6B and 6C).

**Fig 5:** RT-PCR validation of the intestinal (A) interleukin-4 (*IL-4*), (B) interleukin-10 (*IL-10*), (C) interleukin-18 (*IL-18*), (D) interferon-γ (*IFN-γ*), (E) superoxide dismutase 1 (*SOD1*), (F) glutathione peroxidase 1 (*GPx1*), and (G) *occludin* genes in NZW rabbits. *P < 0.05, **P < 0.01 and ***P < 0.001 vs. control. ^+++^*P* < 0.001 vs. NZW+βG_0.25_. Statistical analysis was performed using one-way ANOVA and Tukey's post hoc test for multiple comparisons.

**Fig 6:** RT-PCR validation of the splenic (A) interleukin-1beta (*IL1β*), (B) interleukin-6 (*IL-6*), and (C) inducible nitric oxide synthase (*iNOS*) genes in NZW rabbits. Statistical analysis was performed using one-way ANOVA and Tukey's post hoc test for multiple comparisons.

In APRI breed both 0.25 and 0.5 β-glucan treated groups showed no significant effect on expression levels of intestinal *IL-4*, *IL-6*, *IL-18*, and *IFN-γ* genes (Fig 7A, 7B, 7C and 7D) as well as splenic *IL-1β*, *IL-6*, and *iNOS* (Fig 4). However, in comparison with control, 0.5 β-glucan treated group shows significant upregulation (*P* < 0.001) of both *SOD1* (Fig 3E) and *GPx1* (Fig 7F) mRNA expression, while 0.25 β-glucan treated group showed significant increases (*P* < 0.05) in *GPx1* expression. The 0.5 β-glucan treated group showed significant increases (*P* < 0.05) in intestinal *occludin* expression in comparison with control (Fig 7G).

**Fig 7:** RT-PCR validation of the intestinal (A) interleukin-4 (*IL-4*), (B) interleukin-10 (*IL-10*), (C) interleukin-18 (*IL-18*), (D) interferon-γ (*IFN-γ*), (E) superoxide dismutase 1 (*SOD1*), (F) glutathione peroxidase 1 (*GPx1*), and (G) *occludin* genes in APRI rabbits. *P < 0.05 and ***P < 0.001 vs. control. ^+++^*P* < 0.001 vs. APRI+βG_0.25_. Statistical analysis was performed using one-way ANOVA and Tukey's post hoc test for multiple comparisons.

Splenic mRNA expression of *IL-1β*, *IL-6*, and *iNOS* revealed no significant changes in comparison with control APRI rabbits (Fig 8A, 8B and 8C).

**Fig 8:** RT-PCR validation of the splenic (A) interleukin-1beta (*IL-1β*), (B) interleukin-6 (*IL-6*), and (C) inducible nitric oxide synthase (*iNOS*) genes in APRI rabbits. Statistical analysis was performed using one-way ANOVA and Tukey's post hoc test for multiple comparisons.

## Discussion

Dietary β-glucan administration brought some improvements in animal development and health status [24–26]. Also, β-glucan is considered as an alternative to antibiotics and improves the survival and performance of broilers [27]. In the current study, β-glucan oral administration improved growth performance of NZW and APRI rabbits. Increased efficiency by the nutritional supplement of yeast β-glucan in growing rabbits can lead to increased digestibility and absorption of feedstuffs [28,29]. In addition, improved intestinal health was revealed to increase the villus height, reflecting improved growth efficiency. [30]. In agreement with the current study, Shehata et al [29], Ezema and Eze [31], Bhatt et al [32], and El-Badawi et al [33] found enhancement in BWG and FCR of rabbits administrated with *S*. *cerevisiae* and probiotic.

Some studies support the idea of using prebiotics for increasing the length of the intestinal villus and enhancing immunity [34,35]. Also, this leads to better nutrient absorption, and consequently increases body weight [36]. The enhanced villi height to crypt depth, which would permit higher nutrient intake, may explain enhanced growth efficiency as a response to β-glucans [10,37] and improved intestinal barrier function [38]. Seyidoglu and Peker [39] demonstrated significant increases in thickness of the mucosa, villus heights, crypt depths, and gland depths in rabbits fed diets administrated with yeast that contains β-glucan. A high V/C ratio indicates sufficiently matured and functionally active epithelial cells [40]. In this study, the longest villi values for duodenum were recorded for 0.5 β-glucan, followed by 0.25 β-glucan for both breeds and reflects the absorptive capacity of the intestine.

The present study detected increases of white pulp areas by 0.25 G β-glucan, which reflect on the increase of rabbit immunity. Increased fatty acid utilization due to β-glucan treatment in high fat diet fed mice has been stated by Miyamoto et al [41] and led to a decreased glycogen depletion rate and increased glycogen accumulation in the liver and muscle [42]. Xu et al [43] observed a significant increase in non-esterified fatty acids’ concentration in β-glucan feeding rats, which indicates that β-glucan improves muscle quality due to the increased availability of glycogen. Interestingly, our results showed the significant increase of fiber cross-sectional area of pectoral muscles in 0.5 β-glucan groups. Moreover, glycogen areas were higher in 0.5 G β-glucan of NZW breed and 0.25 β-glucan of APRI breed owing to the higher proportion of high glycogen muscle fibers compared to low glycogen muscle fibers. Therefore, β-glucan could improve the meat quality of rabbits.

Concerning the biochemical findings, ElSawy et al [24] reported that oral administration of yeast β-glucan did not alter serum protein, albumin, and globulin of chicks in comparison with control chicks. Belhassen et al [44] reported that dietary administration of *S*. *cerevisiae* did not alter blood parameters of growing rabbits. The increased uric acid levels in β-glucan-administrated groups may be due to enhancement of purine metabolism and not due to increased kidney function because urea and creatinine levels did not have any changes compared with control.

IL-18 operates to induce a Th1-mediated reaction after exposure to a pathogen in association with IL-12 [45]. An initial increase in intestinal IL-18 gene expression was observed in an unchallenged study on day 7 due to dietary β-glucan, followed by a downregulation on day 14. These findings were consistent with our research, which revealed that the expression of intestinal *IL-18* in NZW rabbit treated with 0.25 and 0.5 β-glucan was considerably upregulated with respect to the control group. IL-18 is an IL-1 family cytokine that has been proposed to promote barrier function in the intestine that improved the gut health against pathogens [46]. In a subsequent research, the expression of IL-18 in birds ' jejunums fed the β-glucan diet was improved [47].

Our outcome shows that there is no important impact on the expression levels of intestinal interleukin-4 (*IL-4)*, *IL-10*, and splenic *IL-6* in separate treatment groups and that the amount of expression of splenic *IL1β*, *IL-6*, and inducible nitric oxide synthase (*iNOS*) in NZ and APRI rabbits shows no important distinction in the control group. The proinflammatory cytokine IL-1 secretion is enhanced by β-glucan [48]. Contradictory information was gathered in mammals where concentrations of IL-6 and TNF-α in β-glucan-fed pigs subjected to lipopolysaccharide decreased relative to their controls [49]. Similar outcomes were noted where intramuscular injection of β-glucan in Wistar rats blocked TNF-α, IL-1β, and IL-6 elevations observed in the control group following sepsis-induced lung injury [50].

When exposed to antigens or chemotactic agents, macrophages start to build iNOS. This enzyme contributes to the development of nitric oxide that then binds to toxic derivatives with superoxide anions, allowing macrophages to skillfully destroy a few kinds of pathogens [51]. Our outcome showed that there were no changes in the splenic iNOS expression rate of mRNA in both NZW and APRI. Cox et al [52] They found no important variations in the rate of expression of the iNOS gene.

Cellular GSH is an essential cellular antioxidant molecule that aids in scavenging of radical species or involvement in antioxidant enzyme catalyzed responses such as GPx [53]. Also, SOD is a critical antioxidant enzyme that protects the cells from the harmful effects of superoxide anion radical [54]. Pretreatment with melatonin or β-D-glucan lowered the harm caused by acetaminophen-induced hepatotoxicity by decreasing oxidative pressure and growing antioxidant activity of GPx, SOD, and catalase (CAT), because melatonin or β-glucan are recognized as free-radical scavengers [55].

Tight junctions consist of at least three types of transmembrane proteins: *occludin*, claudins, and molecules of junctional adhesion. *Occludin* and the family of claudins are the most significant elements of epithelial barrier function in the intestine [56]. Results also indicated that β-glucan upregulated the expression of the intestinal *occludin* mRNA, especially at 0.5 β-glucan [38]. β-glucan upregulated intestinal *occludin* mRNA has anti-inflammatory and antioxidant characteristics [57].

## Conclusion

Dietary immunomodulators such as yeast β-glucan attract considerable attention because they promote indirect development by enhancing immunocompetence in food animals. Here, β-glucan significantly improved villi dimensions, splenic lymphoid diameter, muscular fiber diameter, and muscular glycogen areas. Regarding the breed type, NZW rabbits showed better growth performance than APRI rabbits as represented in the final body weight total daily gain, feed consumption, and total feed conversion ratio. However, carcass traits did not show any significant differences in both rabbit breeds. Oral administration of β-glucan in rabbits will minimize the use of antibiotics, thereby reducing the possible occurrence of drug resistance in bacteria.

## Supporting information

S1 File Raw data of RT-PCR in NZW. (PZF)

S2 File Raw data of RT-PCR in APRI. (PZF)
